The article "PDZ-containing 1 acts as a suppressor of pancreatic cancer by regulating PTEN phosphorylation" was retracted in 2018. Reasons: errors in the data; errors in the images; errors in the text.

# PDZ-containing 1 acts as a suppressor of pancreatic cancer by regulating PTEN phosphorylation

**DOI:** 10.18632/oncotarget.20552

**Published:** 2017-08-24

**Authors:** Qiang Ma, Xiuxiu Wu, Jing Wu, Huanwen Wu, Ying Xiao, Lili Wang, Zhiyong Liang, Tonghua Liu

**Affiliations:** ^1^ Department of Pathology, Peking Union Medical College Hospital, Chinese Academy of Medical Sciences and Peking Union Medical College, Beijing 100730, P. R. China; ^2^ Department of Respiratory Medicine, Peking Union Medical College Hospital, Chinese Academy of Medical Sciences and Peking Union Medical College, Beijing 100730, P. R. China; ^3^ Department of Medical Imaging, Beijing Huairou Hospital, University of Chinese Academy of Science, Beijing, 101400, P.R. China

**Keywords:** pancreatic cancer, prognosis, PDZK1, PTEN phosphorylation, suppressor

## Abstract

Phosphorylation is a recently established cause of phosphatase and tensin homolog (PTEN) gene inactivation, which leads to defect tumour-suppressor function. In pancreatic cancer, this phenomenon has not been reported. Based on database and clinical sample analyses, we found that PTEN phosphorylation occurs in pancreatic ductal adenocarcinoma patient tissues and cell lines, and we aimed to find a method for dephosphorylation. PDZ-containing 1 (PDZK1), a tumour-associated protein that shares its PDZ-binding sequence with the carboxyl-terminal domain of PTEN, was significantly down-regulated in pancreatic cancer as compared to adjacent non-tumour tissues. *In vitro*, PDZK1 overexpression reversed the proliferation and migration abilities of pancreatic cancer cells and led to significantly decreased PTEN phosphorylation and AKT phosphorylation by interacting with wild-type PTEN. In addition, a transcription factor-activation assay supported that PDZK1 overexpression enhanced the anti-oncogene function of PTEN by regulating the activities of its downstream transcription factors, including p53, NF-κB, and FOXO1. *In vivo*, nude mice stably over-expressing PDZK1 had lower tumour weights and volumes and showed significantly down-regulated PTEN phosphorylation in xenograft tumour tissues as compared to the control group. Moreover, low PDZK1 expression strongly correlated with advanced stage and poor prognosis of patients with pancreatic ductal adenocarcinoma. In conclusion, our study elucidated the tumour-suppressor role of PDZK1 in pancreatic cancer through down-regulating PTEN phosphorylation, and established PDZK1 as a potential novel prognostic marker for pancreatic cancer.

## INTRODUCTION

Pancreatic ductal adenocarcinoma (PDAC) is one of the most aggressive and deadly malignancies. Despite an improving understanding of its biology and pathogenesis, contemporary treatment regimens are still lacking in terms of efficacy [1]. Data from recent studies have shown that the occurrence and development of various human tumours are related to the inactivation of tumour-suppressor genes [2–5]. The tumour-suppressor gene phosphatase and tensin homolog (PTEN) regulates a variety of signal-transduction pathways, including the PI3K/Akt pathway, critical to cellular apoptosis, adhesion, and mobility [2]. Loss of PTEN function is common in many tumour types. For example, PTEN is frequently inactivated in gastric cancers because of genetic or epigenetic changes, such as mutations, loss of heterozygosity, promoter hypermethylation, or microRNA dysregulation [6–11]. Recent results have suggested phosphorylation modification of PTEN, involving residues Ser380, Thr382, and Thr383, as a new mechanism of PTEN inactivation in gastric cancer, which may ultimately result in loss of tumour-suppressor function and increased cancer susceptibility [2]. However, the phosphorylation modification and methods for reversing PTEN phosphorylation as a therapeutic option have not been reported in pancreatic cancer.

Structurally, the carboxyl terminal of PTEN has a PDZ-binding motif (residues I400-T401-K402-V403-COOH). PDZ domains are the most abundant protein–protein interaction domains in metazoans. By specific binding to short C-terminal sequences of their ligand proteins, they assemble protein networks and signalling complexes and assist in the targeting and retention of interacting proteins at specialized compartments in the cell. For example, Yao *et al.* found that the PDZ protein can suppress EGF-induced proliferation of breast cancer cells by inhibiting EGFR phosphorylation and blocking EGFR downstream signalling in the cancer cells [12]. PDZK1 (PDZ domain-containing 1) is a type of PDZ domain protein that is expressed at the apical border of epithelial cells in the kidneys, liver, gastrointestinal tract, and pancreas. Owing to its multiple PDZ domains, it can simultaneously bind several ligand proteins and play an important role in molecular regulation [13]. As previously reported, mucins have C-terminal sequences typical of PDZ-domain-binding proteins, exhibit strong PDZK1 binding, and play a specific role in stabilizing Muc3 in the apical membrane of small intestinal enterocytes. Some cancer studies have confirmed that abnormal expression of PDZK1 has been found in several types of tumors, such as renal cell carcinoma, breast cancer, and ovarian cancer, and involved in regulating cancer growth, metastasis and drug resistance by different mechanism [14]. For example, PDZK1 overexpression enhances epidermal growth factor receptor (EGFR)-stimulated MEK/ERK1/2 signalling and IGF-induced Akt phosphorylation in breast cancer [15]. As another example, PDZK1 inhibits the development and progression of renal cell carcinoma by suppression of SHP-1 phosphorylation [14]. However, whether PDZK1 could reverse the malignant phenotype via dephosphorylating PTEN in tumour cells was unknown. In brief, the understanding of the role of PDZK1 in the occurrence and development of tumours is far from complete, especially in pancreatic cancer research.

Therefore, the aim of the present study was to determine whether PTEN phosphorylation occurs in pancreatic cancer tissues from patients with PDAC and pancreatic cancer cell lines. Furthermore, we evaluated whether PDZK1 could reverse the malignant phenotype of pancreatic cancer via dephosphorylating PTEN using *in vitro* and *in vivo* experiments, in an effort to identify the mechanisms of pancreatic carcinogenesis.

## RESULTS

### PTEN phosphorylation is observed in PDAC patient tissues and cell lines

To identify PTEN mutations in different tumour types, we performed an integrated analysis via the cBioPortal and TCGA databases. Overall, among the tumour types examined, PTEN showed the lowest mutation rate in pancreatic cancer (Table 1), with a mutation rate of only 8% (Figure 1A). Next, PTEN mRNA expression levels in normal pancreatic and pancreatic cancer tissues were analysed using the TCGA database. PTEN mRNA expression was not significantly different between normal and cancer tissues (*P* = 0.218; Figure 1B). However, in pancreatic cancer tissues (n = 19), PTEN protein expression was significantly down-regulated (*P* < 0.0001; Figure 1C) as compared to normal pancreatic tissues (n = 6), based on data deposited in the Human Protein Atlas Database. These data may reflect a new mechanism of PTEN inactivation in pancreatic cancer. Next, we detected p-PTEN expression in pancreatic tissues from 15 patients with PDAC by IHC staining. p-PTEN was expressed mainly in the pancreatic ductal cells, and p-PTEN expression was higher in cancer than in adjacent normal tissues (*P* = 0.013; Figure 1D). To validate the phenomenon of PTEN phosphorylation, western blot and immunofluorescence analyses were used to determine the degree of PTEN phosphorylation in 3 pancreatic cancer cell lines. In addition, PTEN mRNA expression levels were detected by RT-PCR. Western blot and immunofluorescence results confirmed that the phosphorylation modification occurred in all 3 cell lines, and PTEN phosphorylation in AsPC-1 cells was higher than that in the MIAPaCa-2 and PANC-1 cell lines. The PTEN phosphorylation level was consistent with the mRNA expression level (Figures 1E–1G). These results confirmed that PTEN phosphorylation occurs in PDAC patient tissues and cell lines.

**Table 1:** Frequency of PTEN alteration in various malignancies

STUDY NAME	ALTERED	STUDY NAME	ALTERED
Uterine Corpus Endometrial Carcinoma (TCGA, Provisional)	67.40%	Esophageal Carcinoma (TCGA, Provisional)	7.60%
Glioblastoma Multiforme(TCGA, Provisional)	41%	Colorectal Adenocarcinoma (TCGA, Provisional)	6.80%
Glioblastoma(TCGA, Nature 2008)	37.40%	Ovarian Serous Cystadenocarcinoma (TCGA, Provisional)	6.80%
Glioblastoma(TCGA, Cell 2013)	30.60%	Liver Hepatocellular Carcinoma (TCGA, Provisional)	6.60%
Prostate Adenocarcinoma(TCGA, Provisional)	21.50%	Head and Neck Squamous Cell Carcinoma (TCGA, Provisional)	6.20%
Uterine Carcinosarcoma(TCGA, Provisional)	21.40%	Colorectal Adenocarcinoma (TCGA, Nature 2012)	6.10%
Merged Cohort of LGG and GBM (TCGA, Cell 2016)	17.50%	Brain Lower Grade Glioma (TCGA, Provisional)	5.70%
Prostate Adenocarcinoma(TCGA, Cell 2015)	17.40%	Breast Invasive Carcinoma (TCGA, Nature 2012)	5.60%
Lung Squamous Cell Carcinoma(TCGA, Provisional)	16.90%	Bladder Urothelial Carcinoma (TCGA, Nature 2014)	5.50%
Skin Cutaneous Melanoma(TCGA, Provisional)	15%	Kidney Renal Clear Cell Carcinoma (TCGA, Provisional)	5.10%
Cervical Squamous Cell Carcinoma and Endocervical Adenocarcinoma(TCGA, Provisional)	13.60%	Kidney Renal Clear Cell Carcinoma (TCGA, Nature 2013)	4.50%
Stomach Adenocarcinoma(TCGA, Provisional)	12%	Lung Adenocarcinoma (TCGA, Nature 2014)	3%
Lung Squamous Cell Carcinoma(TCGA, Nature 2012)	11.20%	Lung Adenocarcinoma (TCGA, Provisional)	3%
Stomach Adenocarcinoma(TCGA, Nature 2014)	11.10%	Kidney Renal Papillary Cell Carcinoma (TCGA, Provisional)	2.50%
Kidney Chromophobe(TCGA, Cancer Cell 2014)	10.80%	Mesothelioma (TCGA, Provisional)	2.30%
Breast Invasive Carcinoma(TCGA, Cell 2015)	10.70%	Head and Neck Squamous Cell Carcinoma (TCGA, Nature 2015)	2.20%
Kidney Chromophobe(TCGA, Provisional)	10.60%	Pancreatic Adenocarcinoma (TCGA, Provisional)	2%
Sarcoma(TCGA, Provisional)	9.90%	Papillary Thyroid Carcinoma (TCGA, Cell 2014)	1.50%
Breast Invasive Carcinoma(TCGA, Provisional)	9.30%	Thyroid Carcinoma (TCGA, Provisional)	1.50%
Pan-Lung Cancer(TCGA, Nat Genet 2016)	8.90%	Pheochromocytoma and Paraganglioma (TCGA, Provisional)	1.20%
TCGA data for Esophagus-Stomach Cancers (TCGA, Nature 2017)	8.70%	Acute Myeloid Leukemia (TCGA, Provisional)	1.10%
Cholangiocarcinoma (TCGA, Provisional)	8.60%	Acute Myeloid Leukemia (TCGA, NEJM 2013)	1%
Lymphoid Neoplasm Diffuse Large B-cell Lymphoma (TCGA, Provisional)	8.30%	Testicular Germ Cell Cancer (TCGA, Provisional)	0.70%
Ovarian Serous Cystadenocarcinoma (TCGA, Nature 2011)	7.90%	Adrenocortical Carcinoma (TCGA, Provisional)	0%
Bladder Urothelial Carcinoma (TCGA, Provisional)	7.90%	Thymoma (TCGA, Provisional)	0%

**Figure 1:** Occurrence of PTEN phosphorylation in PDAC patient tissues and cell lines PTEN mutations in 185 patients with PDAC included in the TCGA database were analysed **(A)**, and PTEN mRNA expression was analysed in normal pancreatic tissue and pancreatic cancer tissue from TCGA database **(B)**. PTEN protein expression level in normal pancreatic tissues (n = 6) and pancreatic cancer tissues (n = 19) from the Human Protein Atlas Database are shown **(C)**. The expression of p-PTEN in surgical samples of 15 patients with PDAC was determined by IHC **(D)**. PTEN phosphorylation was detected in the pancreatic cancer cell lines PANC-1, AsPC-1, and MIAPaCa-2 by western blotting and IF, and PTEN mRNA expression levels were detected by RT-PCR **(E-G)**.

### PDZK1 is associated with malignant phenotype of pancreatic cancer

We explored the PDZK1 expression level in pancreatic cancer using tumour and adjacent non-tumour tissues from the Human Protein Atlas Database. PDZK1 expression was significantly reduced in tumour versus non-tumour tissues (*P* = 0.027; Figure 2A). Multiple microarray analyses suggested that down-regulation of PDZK1 is very common in pancreatic cancer (Figure 2B). To explore the functions of PDZK1 in pancreatic cancer, GO analysis was performed. The results revealed that PDZK1 is mainly involved in regulating cell proliferation (Figure 2C). As tumour occurrence is followed by proliferation and migration, we further investigated the relationship of PDZK1 expression with cell proliferation and metastasis in patients with PDAC, using Gene Set Enrichment Analysis (GSEA). The PDAC patients from the TCGA dataset were divided into high and low PDZK1 expression groups according to median expression level, and correlations with gene sets driving cell proliferation and metastasis were analysed. As shown in Figures 2D-2F, the gene sets were highly enriched in the group with low PDZK1 expression (FDR < 0.05), suggesting that low PDZK1 expression positively correlates with the malignant cell phenotype.

**Figure 2:** PDZK1 is down-regulated in pancreatic cancer and is associated with malignant phenotype PDZK1 expression levels were analysed in pancreatic cancer and normal pancreatic tissues from the Human Protein Atlas Database **(A)**. The expression level of PDZK1 was analysed on the basis of data from multiple microarrays **(B)**. PDZK1 function was analysed on the basis of GO analysis **(C)**. Patient data from the TCGA database were divided into PDZK1-high and -low expression groups, and GSEA was used for enrichment analysis of gene sets related to proliferation, invasion, and migration **(D-F)**.

### PDZK1 overexpression suppressed the proliferation and migration of pancreatic cancer cells

Next, the ability of PDZK1 to modulate pancreatic cancer cell proliferation and migration was analysed *in vitro*. PDZK1 overexpression and knockdown plasmids were constructed and were transfected into MIAPaCa-2 and PANC-1 cells. Western blot analysis confirmed that PDZK1 expression was successfully knocked down and effectively overexpressed in PDZK1 shRNA- and pcDNA 3.0-PDZK1-transfected MIAPaCa-2 and PANC-1 cells, respectively, as compared to cells transfected with the respective empty vectors (Figure 3A and 3B). A CCK-8 assay was used to investigate the role of PDZK1 in cell proliferation. Overexpression of PDZK1 significantly inhibited proliferation in both cell lines studied (*P* < 0.05; Figures 3C and 3D).

**Figure 3:** Effects of stable PDZK1 knockdown and overexpression on proliferation and migration abilities of pancreatic cancer cells *in vitro* PDZK1 was stably overexpressed or knocked down in MIAPaCa-2 **(A)** and PANC-1 **(B)** cells. The proliferative capacity was measured by CCK-8 assays at different time points (24 h to 96 h) **(C** and **D)**. Wound-healing assays were used to evaluate the migration of MIAPaCa-2 and PANC-1 cells **(E** and **F)**. Cells were photographed 0, 12, and 24 h after wounding. Additionally, Transwell assays were performed to evaluate the migration properties of MIAPaCa-2 and PANC-1 cells **(G)**. *p < 0.05; **p < 0.01.

In wound-healing assays, relative narrower distance was observed in PDZK1 knockdown group at 24 hours, while relative wider distance was observed in PDZK1 overexpression group, results revealing that PDZK1 overexpression drastically delayed wound healing (*P* < 0.05; Figures 3E and 3F) in MIAPaCa-2 and PANC-1 cells compared to the respective empty-vector groups. Similarly, in Transwell assays, PDZK1 knockdown group has more cells traversed the membrane compared to empty vector groups, while less cells were observed in PDZK1 overexpression group (*P* < 0.05; Figure 3G), results suggesting that PDZK1 overexpression obviously inhibited cell migration in both cell lines compared with the empty vector groups. In brief, above results authenticated that upregulation of PDZK1 significantly inhibited motility in MIAPaCa-2 and PANC-1 cells.

### PDZK1 inhibits the malignant phenotype of pancreatic cancer cells *in vitro* by dephosphorylating PTEN

Because the carboxyl-terminal domain of PTEN contains a PDZ-binding motif (residues I400-T401-K402-V403-COOH), we investigated whether PDZK1 could regulate PTEN phosphorylation by interacting with PTEN. The PDZK1 expression plasmid was transfected at different concentrations into AsPC-1 cells, which show high PTEN phosphorylation. PTEN phosphorylation decreased gradually with increasing expression of PDZK1 (Figure 4A). Next, PDZK1 was steadily overexpressed or knocked down in MIAPaCa-2 and PANC-1 cells; PTEN phosphorylation was obviously decreased in the PDZK1 overexpression groups (Figure 4B and 4C). Protein–protein interaction (PPI) analysis was performed to investigate the effect of PTEN dephosphorylation on downstream PTEN effectors. Proteins that interacted with PTEN included SLC9A3R1, PIK3CA, PIK3CB, PIK3CD, AKT1, UBC, TP53, JUN, PTK2, and PDGFR. Statistical analysis of the numbers of protein nodes revealed that proteins involved in the phosphatidylinositol 3-kinase (PI3K)/AKT signalling pathway (AKT1, TP53, and PI3K family members) were significantly represented in the PPI network core (Figure 4D and 4E). Constitutive activation of PI3K/AKT signalling promotes the proliferation of various cancers, including pancreatic cancer, while inactivation of this pathway suppresses tumour proliferation, migration, and invasion [16, 17]. Reduced PTEN expression indirectly stimulates PI3K-AKT-mTOR activity, thereby contributing to oncogenesis in humans [18]. To verify the effect of PDZK1 overexpression on downstream effectors in the PI3K/AKT signalling pathway, PDZK1 or PDZK1-shRNA plasmid were transfected into PANC-1 cells, the expression level and phosphorylation of AKT were detected by western blotting. The results revealed that PDZK1 overexpression reduced the degree of AKT phosphorylation (Figure 4F). The activities of the downstream transcription factor (TFs) of PI3K-AKT pathway, NF-κB, p53, and FOXO1, were studied by using a TF-activation profiling plate array with nuclear extracts of pancreatic cancer cells. PDZK1 overexpression increased the p53 and FOXO1 activities, while it significantly decreased the activity of NF-κB (Figure 4G), providing indirect evidence that PDZK1 enhances the anti-oncogene function of PTEN via blocking PTEN phosphorylation.

**Figure 4:** PDZK1 inhibits pancreatic cancer malignant phenotype *in vitro* by PTEN dephosphorylation The PDZK1 expression plasmid was transfected into AsPC-1 cells at different concentrations, and PTEN phosphorylation was detected by western blotting **(A)**. PDZK1 was stably overexpressed or knocked down in MIAPaCa-2 and PANC-1 cells, and PTEN phosphorylation was detected by western blotting **(B** and **C)**. The PPI network was created using the STRING dataset, and the numbers of nodes in the network were counted **(D** and **E)**. The expression level and phosphorylation of Akt were detected by western blot **(F)**. Activities of the transcription factors NF-κB, p53, and FOXO1 were detected by employing a TF-activation plate array with PANC-1 cells **(G)**.

Next, in order to confirm whether the PTEN dephosphorylation regulated by PDZK1 is achieved by interaction with PTEN, PTEN-*wt* and PTEN-*mt* plasmids were respectively transfected into PANC-1 cells with steadily expressing PDZK1, as well as negative control PANC-1 cells. In PANC-1 cells overexpressing PDZK1, the degree of PTEN phosphorylation was significantly decreased after transfection with the PTEN-*wt* plasmid, but not the PTEN-mt plasmid, suggesting that PDZK1 regulated PTEN phosphorylation by interacting with PTEN-*wt* (Figure 5A). Additionally, to investigate whether the tumor suppressor function of PTEN depends on PDZK1, PTEN-wt, PTEN-wt and PDZK1 plasmids were respectively transfected into PANC-1 cells with low endogenous PTEN expression. We found that PTEN-*wt*, when co-expressed with PDZK1, inhibited the proliferation and migration of PANC-1 cells. These phenotypic changes were not observed in PANC-1 cells only transfected with PTEN-*wt* plasmids (Figures 5B-5D). In all, co-expression of PDZK1 and PTEN-*wt* can reduce the level of PTEN phosphorylation and increase the tumor suppressor function of PTEN.

**Figure 5:** PDZK1 regulates PTEN phosphorylation via interacting with wild-type PTEN PTEN-*wt* and PTEN-*mt* plasmids were respectively transfected into PANC-1 cells with steadily overexpressing PDZK1, as well as the controlled PANC-1 cells with empty plasmid, and PTEN phosphorylation was detected by western blotting **(A)**. The proliferation, migration, and invasion abilities of PANC-1 cells transfected with both PTEN-*wt* and PDZK1 or only PTEN-*wt* plasmid were analysed **(B-D)**. *p < 0.05; **p < 0.01.

### PDZK1 inhibits pancreatic cancer growth *in vivo* by dephosphorylating PTEN

*In vivo*, MIAPaCa-2 cells steadily expressing PDZK1 or empty-vector transfectants were injected subcutaneously into nude mice. We found that the tumour-growth rate was significantly decreased in nude mice injected with PDZK1-overexpressing cells, resulting in lower tumour weights and volumes than those observed in the control group (Figure 6A and 6B). These findings were in line with our results *in vitro*, showing that PDZK1 inhibited malignant biological behaviour by regulating PTEN phosphorylation. *In vivo*, we further determined the degree of PTEN phosphorylation by IHC analysis, which revealed that PTEN phosphorylation in xenograft tumour tissues from nude mice steadily expressing PDZK1 was significantly down-regulated when compared to the PTEN phosphorylation levels in the control group (Figure 6C and 6D). Collectively, our results confirmed that PDZK1 inhibited pancreatic cancer growth by dephosphorylating PTEN *in vivo*.

**Figure 6:** PDZK1 inhibits pancreatic cancer growth *in vivo* by dephosphorylating PTEN MIAPaCa-2 cells stably expressing PDZK1 and empty-vector transfectants were injected subcutaneously into nude mice, after which the tumour growth rates **(A)** and weights **(B)** were measured. The levels of PDZK1 and PTEN phosphorylation expression were detected by IHC in nude mouse tumour tissues **(C** and **D)**.

### Low PDZK1 expression is associated with advanced stage and poor prognosis for pancreatic cancer

To further elucidate the role of PDZK1 in PDAC pathogenesis and progression, we analysed the expression levels of PDZK1 in PDAC patients with different tumour stages. Data on the clinical stage, survival time, and genetic alterations of 186 patients included in the TCGA database are shown in Figure 7A. First, we investigated the relationship between the PDZK1 expression level and the T, N, and M stages. The PDZK1 expression level was most significantly correlated with the T stage (*P* < 0.0001; Figure 7B), which is closely related to tumour size and cell proliferation, indicating that PDZK1 significantly correlates with tumour cell proliferation in PDAC patients. The PDZK1 expression level decreased with increasing PDAC stage (*P* = 0.023; Figure 7C), and the fraction of low-level PDZK1-expressing tumours was drastically different between stages I and II/III or IV (Figure 7D), indicating a role of PDZK1 expression in PDAC progression. Thus, we further investigated the PDZK1 expression level as a prognostic indicator. The patients were divided into groups with high and low PDZK1 expression according to median expression level, relative to the median. Kaplan–Meier survival analysis showed that the group with low PDZK1 expression had shorter overall survival and disease-free survival than the group with high PDZK1 expression (*P* = 0.017, *P* = 0.04, respectively; Figures 7E and 7F), suggesting that PDZK1 expression might be a prognostic marker for PDAC.

**Figure 7:** The PDZK1 expression level correlates with progression/prognosis of patients with PDAC The clinical stage, survival time, genetic alteration, and PDZK1 expression level of 185 PDAC patients from the TCGA database are presented **(A)**. The relationship between the PDZK1 expression level and TNM stage was analysed **(B)**. The relationships between PDZK1 expression level and clinical stage **(C)**, constituent ratio **(D)** and survival time **(E** and **F)** were analysed using the TCGA database.

### Up-regulation of PDZK1 alters TF-expression profiles in pancreatic cancer cells

Previous data showed that PDZK1 expression alters downstream TF activity regulated by PTEN. Here, we identified some other TFs activated by PDZK1. The 20 TFs with the most significant changes are listed in Table 2. These 20 TFs play important roles in cancer development by regulating the expression of genes involved in cell proliferation, epithelial-mesenchymal transition, differentiation, and survival. Thus, PDZK1 is a multifunctional adaptor protein that is closely associated with TF activity changes.

**Table 2:** Changes in TF activation in PDZK1-overexpressing PANC-1 cells

No.	TF	PDZK1/vector fold change	Up- or down-regulation
1	Brn-3	956.89	UP
2	RNUX	378.87	DOWN
3	SOX2	280.01	DOWN
4	Snail	177.34	DOWN
5	SOX18	174.08	DOWN
6	Stat4	146.69	DOWN
7	NF-κB	136.17	DOWN
8	SOX9	44.23	DOWN
9	Pax3	28.15	DOWN
10	AP1	27.50	UP
11	ROR (RZR)	24.34	DOWN
12	Prox1	23.80	UP
13	SRY	15.59	DOWN
14	Gli-1	15.29	DOWN
15	TCF/LEF	14.73	UP
16	WT1	14.07	UP
17	MZF	13.72	UP
18	EGR	12.29	DOWN
19	Myc-Max	11.57	UP
20	Pbx1	10.81	UP

## DISCUSSION

PTEN is critical for inhibiting cancer cell proliferation, invasion, and migration [19]. PTEN phosphorylation is a post-translational modification recently discovered as a main cause of PTEN inactivation [2]. Studies on PTEN phosphorylation in malignant tumours, especially, pancreatic cancer, are limited. Few reports of methods for reversing PTEN phosphorylation in malignant tumours are available. In this study, we found that PTEN was rarely mutated in pancreatic cancer as compared to other tumour types, and the relative PTEN mRNA expression level was not significantly different between pancreatic normal and cancer tissues. However, the protein expression level of PTEN was significantly decreased in tumour tissues. With this in mind, we considered that PTEN phosphorylation might occur in tumour cells in patients with PDAC. Consistent with this hypothesis, PTEN phosphorylation was found in PDAC patient tissues and pancreatic tumour cell lines. Based on the structure of PTEN, we identified PDZK1, a scaffold protein that can specifically bind to short C-terminal sequences of PTEN. Deep database analysis revealed that PDZK1 is lowly expressed in pancreatic cancer and correlates with tumour malignant phenotype. By PDZK1 overexpression, the malignant cell phenotype was inhibited *in vitro* as well as *in vivo*. Furthermore, we found that the tumour-suppressor role of PDZK1 is mainly accomplished through regulating PTEN dephosphorylation via interacting with PTEN. In addition, PDZK1 enhanced the anti-oncogene activity through altering the activities of tumour-associated TFs, including downstream molecules in the AKT signalling pathway that are suppressed by PTEN.

In gastric cancer tissues, PTEN phosphorylation has been detected at residues Ser380, Thr382, and Thr383, coincident with reduced expression of PTEN, and PTEN phosphorylation is increased in gastric cancer [2, 20]. Yang *et al* [20] reported an average PTEN phosphorylation rate of 44% in gastric cancer tissues. Consistent with these findings, our results showed for the first time that PTEN phosphorylation at residues Ser380 and Thr382/383 was elevated in PDAC compared to normal pancreatic tissue. We studied the ability of PDZK1 to reverse PTEN phosphorylation in this study. While PDZK1 has 4 PDZ domains and can specifically bind to short C-terminal sequences of PTEN, aberrant PDZK1 expression has been reported in malignant tumours, and PDZK1 is closely related to tumourigenesis. For example, PDZK1 is up-regulated in carcinomas and interacts with the multidrug resistance-associated protein cMOAT (MRP2) [21]. The relationship between PDZK1 overexpression and drug-resistant phenotype has been confirmed in multiple myeloma [22] and breast cancer [23]. In breast cancer, abnormal expression of PDZK1 enhanced cell proliferation in the presence or absence of 17β-oestradiol, potentially through an increase in c-Myc expression. PDKZ1 also interacts with the Src/ER-α/epidermal growth factor receptor (EGFR) complex and enhances EGFR-stimulated MEK/ERK1/2 signalling [15]. In contrast, in this study, we found that the expression level of PDZK1 was significantly decreased in pancreatic cancer, and low PDKZ1 expression correlated with tumour progression. PDZK1 overexpression strongly suppressed pancreatic cancer cell proliferation and migration. These findings may be explained by previous data showing that PDZK1 overexpression causes decreased PTEN phosphorylation and increased PTEN expression. Although several interaction proteins with PDZK1 have been reported [14, 15, 21], there is no information available on its inactivation reasons in tumors. Perhaps hypermethylation of promoter, genetic mutations, and protein post-translational modifications are possible cause of PDZK1 deactivation. Hence, further research will be needed to find the mechanisms of PDZK1 gene inactivation.

As for the downstream mechanism, we constructed a PPI network using the STRING database. According to the node numbers, the PI3K/AKT signalling pathway may play an important role in this network. As previously reported, the AKT signalling pathway is excessively activated in some tumour cell types. For example, PTEN inactivation in gastric carcinogenesis results in the activation of the PI3K/AKT pathway and promotes cell survival [2, 20], and this phenomenon extends to pancreatic cancer [24]. Abnormal activation of AKT promotes cancer progression. In this study, we found that PDZK1 overexpression not only decreased AKT phosphorylation, but also significantly decreased the TF activity of NF-κB, while enhancing the activities of p53 and FOXO1, which are downstream effectors in the AKT signalling pathway. This may be one of the key mechanisms by which PDZK1 inhibits the malignant phenotype in pancreatic cancer. These results confirmed that PDZK1 functions as a tumour-suppressor protein in pancreatic cancer. Our findings conflicted with previous data showing that PDZK1 functions as an oncogene in some tumour types. This contradiction may be explained by variable interactions between the PDZ domains and different tumour-associated proteins. For example, the PDZ domain plays an important tumour-suppressive role in cervical cancer by interacting with EGFR and regulating EGFR signalling [25]. To determine whether PDZK1 overexpression decreases PTEN phosphorylation by interacting with PTEN in pancreatic cancer, a wild-type or mutant PTEN expression plasmid were transfected into PANC-1 cells with overexpressed PDZK1. We found that only co-expression of the wild-type PTEN and PDZK1 could significantly decrease PTEN phosphorylation and suppress cell proliferation and migration. Overall, our data show for the first time that PDZK1 expression can decrease PTEN phosphorylation via interaction with PTEN. These findings confirmed that PDZK1, a multifunctional tumour-associated protein, plays different roles in different tumour types by interacting with different proteins.

In conclusion, this study showed for the first time that PTEN phosphorylation at residues Ser380, Thr382, and Thr383 occurs in PDAC patient tissues and cell lines. PDZK1, as a tumour-suppressor gene, can suppress malignant biological behaviours in pancreatic cancer cells by decreasing PTEN phosphorylation and might serve as a prognostic molecular marker for patients with PDAC. Moreover, PDZK1 can decrease the expression level of AKT phosphorylation and alter the activity of TFs in the AKT signalling pathway. However, insight in the molecular mechanisms of PDZK1 is still lacking. In this study, we only confirmed that PTEN is involved in the dephosphorylation regulated by PDZK1; the direct interaction between PDZK1 and PTEN requires further study. In addition, PDZK1-mediated dephosphorylation is only part of the mechanism underlying the suppression of PDAC-dependent malignant behaviour. The molecular mechanism of PDZK1 in pancreatic cancer requires further exploration. To the best of our knowledge, however, this is the first report showing the prognostic value and clinical implications of PDZK1 for patients with PDAC, thus providing an experimental basis for the clinical treatment of this disease.

## MATERIALS AND METHODS

### Database analysis

TCGA data on mRNA (RNA Seq v2) and clinical data from patients with pancreatic cancer were obtained from https://www.synapse.org/ PTEN mutation rates in all human tumour types were downloaded from the cBioPortal database (www.cbioportal.org). IHC-based protein expression data including high-resolution images were viewed and downloaded from the Human Protein Atlas web portal (www.proteinatlas.org), and the sum IOD of images were analysed by ImagePro Plus software (version 6.0; Media Cybernetics, Rockville, MD, USA). The PPI network of PTEN was constructed using the STRING database (STRING; Search Tool for the Retrieval of Interacting Genes, https://string-db.org).

### Patient tissue sampling and ethics statement

The study was approved by the medical ethics committee of the Peking Union Medical College and was conducted in accordance with the approved guidelines. Fifteen paired tumour and adjacent non-tumour tissues were collected from Peking Union Medical College Hospital (Beijing, China). Informed consent for using the clinical specimens was received from each patient.

### Immunohistochemical (IHC) staining

The tissue sections were de-waxed, hydrated, and incubated in citrate buffer for antigen retrieval. Endogenous peroxidase activity was inhibited with 3% H_2_O_2_. Tissue sections were incubated with a rabbit polyclonal anti-PTEN (Phospho-Ser380/Thr382/Thr383) antibody (1:500 dilution, cat no. D155023; Sangon Biotech) at 37°C for 2 h, washed 3 times in phosphate-buffered saline (PBS) for a total of 9 min, incubated with a horseradish peroxidase (HRP)-conjugated anti-rabbit secondary antibody for 20 min at room temperature, and then washed again. The sections were developed using a 3,3′-Diaminobenzidine Tetrahydrochloride (DAB) Substrate Kit (Thermo Fisher Scientific, Waltham, MA, USA) at room temperature for 1–5 min and counterstained with haematoxylin (Sigma-Aldrich, St. Louis, MO, USA). The results were observed by microscopy (IX71; Olympus, Tokyo, Japan) and analysed with Bio Life DP software (version 4.8).

### Cell culture and transfections

The pancreatic cancer cell lines MIAPaCa-2, AsPC-1, and PANC-1 were purchased from the Cell Resource Center of Beijing Xiehe (Beijing, China) and cultured in high-glucose Dulbecco's modified Eagle's medium (DMEM; Cell Resource Center of Beijing Xiehe) or Roswell Park Memorial Institute 1640 medium (Gibco, Waltham, MA, USA) supplemented with 10% foetal bovine serum (Thermo Scientific; Waltham, MA, USA) and penicillin (100 U/mL; Cell Resource Center of Beijing Xiehe). The 3 cell lines were cultured in an incubator maintained at 37°C with 5% CO_2_. The expression plasmid pcDNA 3.0-PDZK1, the knockdown plasmid PDZK1-shRNA, PTEN-*wt* plasmid (last four amino acids was ITKV), PTEN-*mt* plasmid(last four amino acids were point-mutated from V to A: ITKA)and the respective empty vectors were preserved in our laboratory. Lipofectamine 2000 (Invitrogen, Carlsbad, CA, USA) was used for transfections, following the manufacturer's protocol. To generate stable knockdown clones, MIAPaCa-2 and PANC-1 cells transfected with the knockdown plasmid were cultured in medium containing 2 μg/ml puromycin for 4 days. To generate stable overexpression clones, MIAPaCa-2 and PANC-1 cells transfected with the expression plasmid were cultured in medium containing 200 μg/ml G418 (Geneticin) for 4 weeks. The PTEN-*wt* and PTEN-*mt* plasmids were co-transfected with pcDNA 3.0-PDZK1 into PANC-1 cells.

### Western blot analysis

Cells were collected and lysed in radio-immunoprecipitation buffer (Beijing CoWin Biotech Co., Ltd., Beijing, China) in the presence of protease inhibitors for 30 min to extract total proteins from cells with stable overexpression or knockdown of PDZK1 and control cells. Protein levels were quantified by bicinchoninic acid assays (Beijing CoWin Biotech Co., Ltd.). Thirty micrograms of protein from each sample was resolved by 10% sodium dodecyl sulphate-polyacrylamide gel electrophoresis (Beijing CoWin Biotech Co., Ltd.). Proteins were transferred to nitrocellulose membranes (Sigma-Aldrich), which were blocked for 1 h in bovine serum albumin blocking buffer (Invitrogen Life Technologies). Subsequently, the membranes were incubated overnight at 4°C with primary antibodies targeting PDZK1 (1:500 dilution, cat no. D154222, Sangon Biotech), PTEN (1:300 dilution, cat no. D261095, Sangon Biotech), p-PTEN (Phospho-Ser380/Thr382/Thr383) (1:500 dilution, cat no. D155023, Sangon Biotech), or GAPDH (1:5000 dilution, cat no. 70699, Abcam), followed by incubation with an HRP-conjugated goat anti-rabbit secondary antibody (1:3000 dilution, cat no. CW0103, Beijing CoWin Biotech) for 1 h at room temperature. Immunocomplexes were detected using an enhanced chemiluminescence kit (Thermo Scientific), and images were analysed using Image J software (version 1.62; National Institute of Health, Bethesda, MD, USA).

### Determination of PDZK1 and PTEN mRNA levels by RT-PCR

AsPC-1, PANC-1, and MIAPaCa-2 cells were harvested, and total endogenous mRNA was isolated using the RNeasy Mini Kit (Qiagen, Hamburg, Germany). RNA was treated with DNase (Qiagen) to eliminate any DNA contamination. Total RNA was reverse-transcribed to cDNA, and the first-strand cDNA was used as a template for real-time PCR. Real-time PCR was carried out using the qPCR Master Plus for SYBR Green I-DTTP (Eurogentec, Belgium) with gene-specific primers in a DNA Engine Opticon 2 system (MJ Research Incorporated, BioRad, Philadelphia, PA, USA). All reactions were run in triplicate. Relative gene expression was quantified using β-actin as an internal control.

### Immunofluorescence assay

Pancreatic cancer cells (AsPC-1, PANC-1, and MIAPaCa-2) were cultured in 6-well plates (2 × 10^5^ cells/well) containing glass coverslips for 24 h. Cells were fixed with 4% paraformaldehyde at room temperature for 15 min, followed by 3 washes with 1× PBS. Next, the cells were treated with 0.5% Triton X-100 for 20 min. The cells were incubated overnight at 4°C with an anti-p-PTEN antibody (1:50 dilution, cat no. D155023; Sangon Biotech), followed by 3 washes with 1× PBS. The cells were incubated with a goat anti-mIgG conjugated with fluorescein isothiocyanate (1:50 dilution, cat no. D155023, Invitrogen) for 60 min, followed by 3 washes with 1× PBS. Cell nuclei were stained with DAPI (Zhongshan GoldenBridge Biotech, Beijing, China) for 5 min. p-PTEN was observed by fluorescence microscopy (IX71; Olympus) and Bio Life DP software. These experiments were repeated at least 3 times.

### Cell proliferation assay

Cells transfected with the PDZK1, PTEN-*wt*, PTEN-*mt* plasmids were plated at a density of 5 × 10^3^ cells/well in 96-well plates and incubated at 37°C with 5% CO_2_. Cell proliferation was assessed every 24 h for 96 h using the CCK-8 kit (Sigma-Aldrich St. Louis, MO, USA), according to the manufacturer's protocol. For each sample, 6 wells were analysed at each time point. The experiments were repeated 3 times.

### Cell migration assay

Cell migration abilities were determined in Transwell and wound-healing assays. Briefly, to determine the migration potential, DMEM containing 10% FBS was added to the lower chambers, and 1 × 10^5^ cells suspended in 200 μl serum-free medium were added to the upper chambers and cultured for 16 h. The cells that had traversed the membrane were stained with crystal violet. The mean number of cells was calculated by five fields randomly under microscope (10×20). For wound-healing assays, cells were plated at a density of 2 × 10^5^ cells/well into 6-well plates and grown to 80% confluence. The cell monolayer was scratched with a 1-ml pipette tip to create a wound and an image was captured immediately (0 h). Migration was observed every 12 h and images of the closing wound were captured at every 12 h with image acquisition software (Bio-Life DP, version 4.8) connected to a phase contrast microscope (CKX41; Olympus). The same visual field was used throughout the experiment. ImagePro Plus software was used to calculate the relative scratch distance as follows: relative scratch distance = wound area/wound height.

### Transcription factor (TF) activation profiling

We utilized a TF Activation Profiling Plate Array Kit user manual (Signosis, Inc.) per the manufacturer's instructions to identify TF activities affected by PDZK1 in PANC-1 cells. Nuclear extract (10 ug) was first incubated with the biotin-labelled probe mix at room temperature for 30 min. Activated TFs were bound to the corresponding DNA-binding probes. After the protein/DNA complexes were isolated from the unbound probes, the bound probes were eluted and hybridized to a plate pre-coated with capture oligos. The captured biotin-labelled probes were detected with streptavidin–HRP and subsequently measured using a chemiluminescence plate reader (Turner microplate multimode, Turner BioSystems).

### Animal experiments

Cells stably transfected with the pcDNA 3.0-PDZK1 and pcDNA 3.0 vectors in exponential growth were harvested, washed twice in PBS, and resuspended in PBS at 6 × 10^7^ cells/ml. The cell suspension (0.1 ml; 6 × 10^6^ cells) was subcutaneously injected into the right flanks of 5- to 6-week-old female BALB/c mice (n = 7/group), which were purchased from Beijing Vital River Laboratory Animal Technology Co., Ltd. and maintained in microisolator cages. Tumour volumes (mm^3^) were measured every 3 days in 2 dimensions, using a calliper. After 4 weeks, the tumours were removed from the mice and weighed. These experiments were conducted according to the International Guidelines for the Care and Use of Laboratory Animals (The United Kingdom Coordinating Committee on Cancer Prevention Research's Guidelines for the Welfare of Animals in Experimental Neoplasia), and were approved by the Institutional Animal Care and Use Committee of Peking Union Medical College.

### Statistical analysis

Data were analysed using SPSS software, version 21.0 (SPSS Inc., Chicago, IL, USA) and GraphPad Prism 5 (GraphPad software Inc., San Diego, CA, USA), and are presented as the mean ± SD from at least 3 independent experiments. TCGA data for paired samples were analysed by paired-sample *t*-testing. Growth curves were analysed using repeated-measures analysis of variance with Fisher's least-significant difference post-hoc test. Data from Transwell and wound-healing assays and IHC staining data for unpaired samples were analysed by independent-samples *t*-testing. The relationship between the PDZK1 expression level and clinical stages was analysed by one-way analysis of variance. A log-rank test for the generated Kaplan–Meier curve was conducted to evaluate the association between the expression level of PDZK1 and survival rate. Overall survival was defined as the time between the first surgery for primary pancreatic cancer and death for any reason. Disease-free survival was defined as the time between the first surgical resection and disease recurrence. *P* < 0.05 was considered to indicate a statistically significant difference between values.
